The article "LSTM-Based Deep Model for Investment Portfolio Assessment and Analysis" was retracted in 2023. Reasons: signs of a paper mill; suspected computer-generated content; unreliable results or conclusions; concerns about the data.

# LSTM-Based Deep Model for Investment Portfolio Assessment and Analysis

**DOI:** 10.1155/2022/1852138

**Published:** 2022-07-07

**Authors:** Haohua Yang

**Affiliations:** College of Letters and Science, University of California, Santa Barbara, CA 93106, USA

## Abstract

In recent years, within the scope of financial quantification, quantitative investment models that support human-oriented algorithms have been proposed. These models attempt to characterize fiat-delayed series through intelligent acquaintance methods to predict data and arrange investment strategies. The standard long short-term memory (LSTM) neural network has the shortcoming of low effectiveness of the fiscal cycle sequence. This work utters throughout the amended LSTM design. The augury result of the neural reticulation was upgraded by coalesce attentional propose to the LSTM class, and a genetic algorithmic program product was formulated. Genetic algorithm (GA) updates the inalienable parameters to a higher generalization aptitude. Using man stock insignitor future data from January 2019 to May 2020, we accomplish a station-of-the-contrivance algorithmic rule. Inferences have shown that the improved LSTM example proposed in this paper outperforms other designs in multiple respect, and it performs effectively in investment portfolio design, which is suitable for future investment.

## 1. Introduction

With the forcible educement of all-inclusive economic and bursal quotations, as the barrier of financial quotations and an important part of the appraise of derivatives, the haleness of the futures mart is more and more important for the entire preservation and quality regulation. Strategy carries a lot of weight nowadays. Premeditated future prices can take the lead at the macrolevel and correct the predictability and power of the macrogovernment. It can also observe and analyze return fluctuations in the future market and further predict future real addresses and macroeconomics. Toby's stretch can more effectively reveal and judge the behavior of macrosavings. The forecast of future price operation is mainly divided into fundamental analysis and technical analysis. Fundamental analysis is to predict future trends based on the business and macrofundamentals of future varieties. For delegates, the occurrence of certain events tends to result in significant fluctuations in the assets being charged. Meanwhile, the loosening of important economic data can also be a major blow to selling trends. Technical analysis assumes that stories are similar or repeatable, through data and elements. Over the years, as technology has progressed and developed, various types of forecasting ideas have been proposed, mainly because of the advent of deep neural networks. This is because of their solid nonlinear fitting ability and powerful nonlinear fitting ability, which are gradually applied to the analysis and prediction of financial asset value [1–7].

The article "LSTM-Based Deep Model for Investment Portfolio Assessment and Analysis" was retracted in 2023. Reasons: signs of a paper mill; suspected computer-generated content; unreliable results or conclusions; concerns about the data.

Stocks are an important part of capital value construction, and the qualification of stock selling is extensible for general macroeconomics, investment institutions, and investors. This characteristic can not only lead to higher feedback from investors but also improve the integration and flexibility of investment. The technology is convenient for investors to buy brass and deliver investment funds at any time. Therefore, the Pillar Market has becoming an ideal place for the community to conduct financial exchanges. There are many alternatives to enhance cumulative market value movements, such as association news and performance, industry work, investor sentiment, social media opinion, and economic factors. The high volatility and insecurity of fund rewards make it a mayoral proposition in fiscal research. Stocks are dangerous property. Predicting stock prices can help investors avoid danger and reform the safety and profitability of stock investing. Therefore, there is an urgent requirement to study stock price forecasting methods to minimize investment risks and improve investment returns, such as the positive intent. Traditional forecasting methods are often difficult to balance the randomness and regularity of changes in holding rates. Thus, more or less failure cases will occur [1]. With the advancement of technology, machine intelligence and deep learning algorithms have been widely used in the field of financial investigation. The authors [2] used shape-preserving vector (SVM) to simulate hoarding rate diversification. The model is characterized by familiar technical indicators, but the selection of indicators is supported by basic experience and has strong objectivity. Balaji et al. [3] have long supported four deep letter shapes, short-term conditional recall network (LSTM), gated controlled recurrent networks (GRU), convolutional neural plexus (CNN), and outermost learning bikes (ELM), predicting S&P stocks. BANKEX index and termination have shown that all complex legend models can produce commendable prediction precision. In modern times, inventory cost forecasting methods based on affected neural networks and informed technologies have been widely utilized to better compensate for the shortcomings of traditional forecasting methods and improve the reliability and fairness of store price forecasting [4] In [5], the authors compared the effectiveness of deep neural plexus (DNN) and shallow neural network (SVM and single-band neural network) in stock divination. The reasoning results have shown that the prediction performance of DNN was significantly better than that of simple neural spider web [6–12].

The article "LSTM-Based Deep Model for Investment Portfolio Assessment and Analysis" was retracted in 2023. Reasons: signs of a paper mill; suspected computer-generated content; unreliable results or conclusions; concerns about the data.

Applying the LSTM model to stock price trend variations, and comparing its prediction results with the harbingers of feedforward neural network (BP) and recurrent neural network (RNN) schemes, we can conclude that the prediction effect of LSTM is more correct than that of BP and RNN. The parameters used in forecasting are limited, and the results of harbingers are not psychological. In addition, the authors [8] proposed the LSTM network example into the prediction of pillar returns, and further obtain the characteristics of the prediction fidelity of the model with different input features. The authors [9, 10] applied the LSTM fashion to the prediction of cumulative reward volatility, and further used its prediction results. Compared with the prediction results of 18 classical models, the LSTM h is validated. The pipeline of our adopted LSTM model is presented in Figure 1.

## 2. Related Work

The work of age series data prediction has a solid affinity with regression analysis in bicycle literature classification methods, and artificial neural networks are considered as effective tools to achieve repeated train prediction [2–14]. This illusory abstract abstracts the main learning content of the lab recently, and reviews the characteristics and shortcomings of each algorithm program in the application of three aspects: the main problem, shape engineering and the touch of machine literature algorithms. Focusing on the main obstacles encountered by current machine learning in hoarding oracles, it analyzes and looks forward from the aspects of token literature, shape engineering, and unmixed scientific model association. The modified Elman neural network model improves the prediction accuracy of existing Elman neural networks for seasonal series data. Experimental inferences show that the inverse model has higher fidelity in predicting fiscal age inheritance. The authors [5] took the lead in granting the application and exploration of the dual-influence dilated neural plexus method in the field of stock index futures forecasting analysis, and explained in detail the composition intention and algorithm program flow of the two dual-weight dilated neural networks. The utility in the response is supported by evidence. Among complete neural networks, repetitive neural networks are a good model for predicting chance sequences. Since the input of a feedforward neural network only turns on the current input, the neurite repeat sequence data is laborious. Feedback neurons can respond to time-varying data of any length. LSTM and GRU are old recurrent neural network formations. The authors [6, 7] applied LSTM to deal with the thirst-alienation stock time series problem and invented a few advanced shape system memory networks that belonged to restricted and imperfect words. The input was customized for training, and the effectiveness of variables was comprehensively analyzed through experiments. form of prediction. The inset results show that the Dobaraka feature system has certain advantages in prediction. The authors [8] employed stacking denoising to extract features from barebones market data and technical indicators of financial measurement trains and use them as inputs to LSTM neural networks to obtain relatively high prediction accuracy. The authors [9, 10] used an unmixed LSTM grid to virtualize financial data and to address long-term dependencies between data, and to study more complex market dynamics, the model introduced an attentional clockwork that made the data important. Sex is predicted differently in different sets and validated more correctly. The authors [11] jointly studied the prediction of delayed sequences implemented by a cascade mechanism, which not only introduced nursing clockwork in the input stage of the decoder but also introduced an attention mechanism in the encoder stage. prophecy. This paper combines the notification mechanism with LSTM to try to improve the implementation of standards in future investment strategies. Genetic algorithms are often used for model parameter tuning. The authors [12] discussed a modified LSTM neural network stock-pointing omen and analysis method based on genetic algorithm rules and tilted three models to Nasdaq, respectively. The experimental results show that compared with the other two methods, the authenticity of the proposed method has been significantly revised in terms of significant capital volatility, and the fundamental trend can also be predicted in the stage of comprehensive stock volatility. In [13–19], the authors proposed the genetic algorithm rules used to solve the proposition of parameter solving to ensure the adjustment of the model divination, and it has been proved that all aspects of the modified shape are better than the single LSTM approach.

The article "LSTM-Based Deep Model for Investment Portfolio Assessment and Analysis" was retracted in 2023. Reasons: signs of a paper mill; suspected computer-generated content; unreliable results or conclusions; concerns about the data.

In recent years, some portfolio examples performed well in predicting supply value settings. The authors [11] adopted autoregressive moving average bifurcations, exponential smoothing models and RNNs to systematically mix models.. The verification results show that the combined model has a reforming effect than the weak wear RNN. The authors [12] used primitive element analysis (PCA), genetic algorithm (GA), and BPNN to predict the capital value, and the problem shows that the accuracy of divination is more accurate. The authors [13] discussed an example of LSTM with overfitting prevention and an example of LSTM-based forecasting framework for supply market indices. Spring shows that the model has good prediction fidelity. The authors [14] combined the LSTM model with various Generalized Autoregressive Conditional Heteroskedasticity (GARCH) criteria to propose an unworn feature selection algorithm.

## 3. Our Proposed Method

The technical indicator is the determined result obtained by saving the source data in an unquestionable flow algorithm program according to the stock data sequence. The stocking data means the processed result is a data sequence. Technical indicators play a far-reaching role in supply market forecasting and analysis and are insightful, specific, and easy to apply in judging the government value of a store. Different technical indicators have different objectives and constraints. When performing stock feature representation, a single technical trader cannot guarantee the comprehensiveness and fairness of feature presentation. Therefore, selecting a variety of typical and easy-to-evaluate technical indicators can correct the complementarity of data and the fidelity of feature representation. In this paper, the forecast table set supported by 16 technical indicators commonly used in the stock market is elaborated in [13]. These indicators fully believe that the trend deviates from the value-hoarding advertisement and can contain most of the later price influencer forecasts.

LSTM can be deemed as a special version of RNN, which solves the problem of exploding gradients and vanishing slopes of RNNs during long-term development. The phenomenon of forgetting is built upon the previous information over time. On the basis of the conventional RNN, LSTM adds a memory to each nerve in the hidden layer, so that the memory information in the time series is controllable, so that the powerful Moses law between data can be inserted more deeply, and the divination is more accurate and reliable. The schematic diagram of the composition of the LSTM storage unit is shown as follows:

(1) $$\begin{array}{c} f_{i}=\sigma \left(W_{j}x_{i}+W_{h}h_{i-1}+b_{j}\right), \end{array}$$

where *W*_(*t* − 1) and *h*_(*t* − 1) are the biased acme of the memorial one and hidden lift in the preceding sense and *S*_*t* and *h*_*t* are the stream state of the reminiscence one and the possession of the unknown basis, respectively. The top-down path f_t, the input reciprocate x_t, and the product are connected to each other to handle the memorial and lightness of previous and stream notifications.

The article "LSTM-Based Deep Model for Investment Portfolio Assessment and Analysis" was retracted in 2023. Reasons: signs of a paper mill; suspected computer-generated content; unreliable results or conclusions; concerns about the data.

The flow chart of the RF-LSTM prediction standard is presented as follows. And the remedial trajectory is as follows. (1) Obtain the stored data, arrange the predicted technical indicators into a feature set, and renormalize the form set. (2) Train a random forest and resample using the bootstrap method. The probability of not being drawn is (1-1/N)N for each example in the source data that specifies self-stamping (OOB) data. (3) For each partition tree, select the corresponding out-of-bag data to rate the out-of-bag data illusion, denoted as errOOB1. (4) Add din interference randomly to all matching features *x* of OOB data, and consider the error of OOB data again, denoted as errOOB2. Assuming that there are *N* woods in the wild wood, the importance calculation formula of feature *x* is as follows:

(2) $$\begin{array}{c} \text{FI}{\text{M}}_{x}=, \end{array}$$

where in (2), FIM is the feature importance score (formation importance measure), and it is reported randomly after increasing. If the authenticity of the OOB data decreases (i.e., err_ob2_ retires), it means that this shape has a huge prestige in the example divination results; that is, the importance is relatively high. (5) Calculate the shape importance, and then sort by importance. (6) According to the analogy out-of-bag error rate of each feature set and form set obtained above, select the feature that is suitable for the last out-of-bag error rate. (7) The culling features are prepared to be input into LSTM for divination, the prediction results are compared with the sample tassel, the cross-entropy failure performance is calculated, and the Adam optimization process is used for moment optimization. (8) Test the exercise method with test data, get the final forecast result, and compare it with the real stock value to induce closing.

Besides the LSTM, the so-called genetic algorithm (GA) is a powerful hunting and optimization method developed based on biological evolution mechanisms such as natural reference and genetic variation. GA imitates the innate biological mobility mechanism. Its scent is a competent, parallel, global search method that automatically learns and accumulates acquaintances about the search room in the search projection. Then, the exploration process is coordinated under the supervision of the successful optimal discharge. The implementation process of genetic algorithm rules is roughly divided into the following steps:

Initialize the population: first, we digest the requirements. The feasible disassembly of the problem is formulated as chromosomes or individuals in the gene compartment

Fitness: fitness is the degree to which an individual dominates the lifespan of a population, as measured by health performance or by an assessment office

Choice: we interpret this as a crisis of further repetition. For example, roulette offers tournament selections

Intersection: it describes how to compose an unaccustomed solution from an existing disintegration, for example, *n*-appointment intersection.

The article "LSTM-Based Deep Model for Investment Portfolio Assessment and Analysis" was retracted in 2023. Reasons: signs of a paper mill; suspected computer-generated content; unreliable results or conclusions; concerns about the data.

Mutation: its examples are the insertion of differentness and novelty into the delivery pool by randomly swapping or closing solutions, such as binary changes.

Since this paper utilizes an atavistic neural network model, the RNN structure of discontinuous neural networks makes them difficult to parallelize. Thus, training repetitive neural networks take a lot of time. Using genetic algorithm rules to tune the parameters of the RNN will further increase the tuning time of the entire model. Therefore, it is very disturbing that the GA rules can converge faster. From the above progress, we can know that the cross-speculator is suitable for merging optimized genes, the change-speculator is responsible for inspecting the whole room extensively, and the selection operator is responsible for selecting solutions with high fitness values. Both crossover and change are unguided. Therefore, choosing a speculator must ensure that the group is moving towards its intended goal. By selecting speculators, individuals with transcendent fitness will have more chances to be eliminated as the parents of the next generation of nests [15]. Based on this, this journal improves the selection and speculation part of the genetic algorithm to accelerate the convergence of the genetic algorithm program. Selection speculators are usually interested in genetic algorithms as roulette selection methods. The old-fashioned roulette selection method aggregates the fitness values of individuals and then normalizes them and then selects the individuals corresponding to the area where the random number becomes the speed number, which is specific to the spinning roulette of the casino. Each special selection opportunity corresponds to its fitness value, and the greater the fitness, the greater the possibility of selection. In order to speed up the convergence, the model in this paper adopts the modified roulette selection method. In the traditional roulette quoting method, since all fitness in a population emergency needs to cross each tempo search, the time complexity of the algorithm depends on the population count *N*, which is O(N) or O(logN). Time entanglement can be reduced to O(1) by leveraging the method supported by conjecture acceptability of roulette selection.

## 4. Experimental Results and Analysis

In order to judge the causal relationship of this journal's approach, the original data studied in this paper came from the Tushare financial data package. Tushare is a free, obvious source python financial data interface package. It can powerfully complete the data collection, cleaning, promotion, and data storage of financial data such as Bitstock and can provide financial analysts with indestructible, clean, and easy-to-analyze different data. The data package contains the information of Shanghai Pudong Development Bank from 2017.04 to 2019.05 for a total of 524 trading days, including 5 sets of transaction data, namely, the starting price of the maid, the meridian market, the final price, the final value, and the workload. 80% of the samples in the relish subset are adjusted as feature selection samples, and 20% of the samples are determined as independent experiments. Forms were chosen to discriminate on an unconstrained test set, and no form-referenced classification oracles were applied as comparative experiments. Build a feature set using culled data. Due to the estimation methods of various other indicators, the shape quantities constructed according to the technical indicators have different value ranges, and the photometric screening is very obvious. Large numerical differences can complicate the optimization of the algorithm's standard parameters, overfitting is slight, and there is a reluctance to the final prediction termination. Therefore, in this paper, Equation (1) is useful to normalize the feature quantities, and the formal components of each girt are regenerated as [-1, 1].

The article "LSTM-Based Deep Model for Investment Portfolio Assessment and Analysis" was retracted in 2023. Reasons: signs of a paper mill; suspected computer-generated content; unreliable results or conclusions; concerns about the data.

In this wallpaper, Anaconda software is the necessary software for building models, data output mainly supports pandas and numpy modules, and example analysis uses Sklearn and keras modules. The value of each parameter in the design is shown in Table 1. For the tempo series, the data in *n* times [*X*(*t* − *n*), *X*(*t* − *n* + 1), ⋯, *X*(*t* − 1), *X*(*t*)] is usually used as a prediction (*t* + 1) chance data input. For stocks, there will be several shape data at time *t*. Therefore, in the case where the management and storage features and models are more accurate, this paper takes a two-dimensional vector of *n* (metric sequence) × *s* (formal data) as input, takes the most ideal feature ⊆ at the origin as the input variable, and the input chance harness is 30 days, with flow days as the product variable. The LSTM die has 4 boosts, i.e., 1 LSTM coping +3 dense layers. When discipline LSTM shape, dropout parameters and consistent stipulation are added to avoid overfitting. Offer degree regulated second-hand chastisement model prediction criteria while rise worn traditionary LSTM prediction propose. Indicated absolute error (MAE), indicated quadratic fallacy (MSE), and root mean square drift (RMSE) were tailored as appraisement metrics to assess the authority of bifurcations. The measurement formulas of the three evaluation indicators are shown in Table 1.

The article "LSTM-Based Deep Model for Investment Portfolio Assessment and Analysis" was retracted in 2023. Reasons: signs of a paper mill; suspected computer-generated content; unreliable results or conclusions; concerns about the data.

According to the RF-LSTM algorithm program to extract features, the hold shape matter musty is shown in Table 1, where the vertical axis is the feature set of the predicted invention of 16 technical indicators, and the horizontal axis is the subject form measure. It can be seen from Table 1 that the importance of OBV, ATR, and ADX is very high, while the importance of other shapes is very serious, all less than 0.1. The decisive ideal shapes ⊂ are OBV, ATR, and ADX. Use OBV, ATR, and ADX to replace the original basic data as training data for modeling, while retaining most of the teaching content contained in the data and the original data expansion is weakened. The results of the supply quotation schemes of different forecasting models are shown in Table 1, with a total of 50 trading days of ups and downs. To validate the fashion of this paper, the shape importance rankings in Table 1 are shown. We sort the graph of reimportance effectiveness and odds and get the predictive inference of RF-LSTM and LSTM. From Table 1, it can be seen that both RF-LSTM and LSTM alone can predict the common trend of postal prices. However, there is a dispersion gap between the predicted termination value and the true value of LSTM, mainly because for repeated training of bursts with report, this feature also contains cry and information redundancy, and the formal lineage of the unmixed model is not thorough, in which eventually, the prediction effect of the noncomposite model is not ideal. The predicted value of the RF-LSTM model is closer to true excellence, the prediction fidelity is higher, and the support rate is improved. On the whole, the fitting effect of the mold is relatively large. It is revealed that when the optimal number of variables is predetermined, the size of the input boost and the number of nodes in the secret layer can be suppressed, the network structure can be simplified, the fork vulnerabilities can be fixed, and the omen importance can be shifted and correct The value wheel can improve the fit.

The prominent price prognosis errors of distinct forecast de facto folks are shown in Table 1. The MAE of RF-LSTM is 14.59%, while the MAE of LSTM is 27.70%. MAE is the standard bright of the unconditional fault between the foreshow advanced and the observed refulgence. The MSE of RF-LSTM is 4.10%, while the MSE of LSTM is 10.81%. MSE is the degradation of the sum of quarrel deviations of the data from the allegiance importance. The greater the degree of goodness, the worse the germination performance. RMSE is the sample-marker deviation of the predicted value versus the observed value (called the residual), which accounts for the degree of dispersion in the sample. When the nonlinearity is suitable, the smaller the RMSE, the more correct. The RMSE of RF-LSTM is 20.24%, while the RMSE of LSTM is 32.78%. As can be seen from Figure 2, the prediction error of the RF-LSTM fork is smaller compared to the conventional LSTM example. The smaller prediction illusion attempts to give fashion a better expression in stock quotes and predictions, with better generality and consistency.

The article "LSTM-Based Deep Model for Investment Portfolio Assessment and Analysis" was retracted in 2023. Reasons: signs of a paper mill; suspected computer-generated content; unreliable results or conclusions; concerns about the data.

## 5. Conclusions

This paper first introduces different methods for future price forecasting and then proposes an improved LSTM-Attention-GA model based on long short-term memory neural network, which combines attention mechanism and genetic algorithm. Then, the experimental method is introduced. The required software and hardware, data acquisition, and processing process are obtained. Finally, the comparative experiments show that the LSTM-Attention-GA model we constructed has achieved the effectiveness of the future investment strategy and solved the problem that the traditional LSTM neural network cannot predict financial time series. Therefore, it is of great significance for the application of neural network models in financial markets.

In the future work, the direction that can be expanded includes mining more and more effective factors; instead, use higher frequency data or even tick-level data for training, because more data will help the model to further explore data features. It also includes how to build a better model to reduce overfitting in training, as well as the problem of slow model training. In addition, the genetic algorithm may also fall into a local optimum instead of obtaining a global optimum. If this is prevented, the situation and how to further improve the prediction effect are also the directions for further research in the future.

## Figures and Tables

**Figure 1:** An example of the basic LSTM for stocking price prediction.

**Figure 2:** The shrinkage speed by varying the number of iterations.

**Table 1:** Parameter tuning correspondence.

Parameter	Meaning	LSTM-A	LSTM-GA
*n*-Step	Time step	12	15
Hidden-size	Hidden neuro number	16	19
MA (*n*)	Shift number	14	17
RS (*n*)	Strong att	7	11
WILLR (*n*)	Weak att	18	21
CCL (*n*)	Long att	23	25

## Data Availability

The data used to support the findings of this study are available from the corresponding author upon request.
